# Research on the Throwing Technique of High-Pole Hydrangea Champion Team in the 12th Students' Games of Guangxi

This article has been retracted.

**DOI:** 10.1155/2022/6422746

**Published:** 2022-04-15

**Authors:** Shijun Xu, Cong Zeng, Pei Yang, Yu Wei

**Affiliations:** ^1^Physical Education College, Guangxi University of Science and Technology, Liuzhou 545006, China; ^2^Sports Department, Liuzhou Institute of Technology, Liuzhou 545006, China; ^3^Liuzhou Sports Bureau, Liuzhou 545006, China

## Abstract

By using the methods of literature, mathematical analysis, and comparative analysis, this study expounds the origin and development history of the culture of Hydrangea and the movement of throwing Hydrangea, studies the representative technical theory of high-pole throwing Hydrangea, and makes a comparative analysis with the angle, speed, and other technical movements of throwing Hydrangea in teaching and training, as well as the trajectory data of the arc top height, circle range, and landing point of the parabola of Hydrangea. This study discusses the technical problems existing in the high shot Hydrangea competition of the two students Games in Guangxi. The research shows that projection technology is the foundation and core element of the survival and development of high-pole throwing Hydrangea; the existing projection technology has a certain positive effect on teaching, but it has shortcomings for high-level training and competition. The research shows that throwing technology is the foundation and core element of the survival and development of high-pole throwing Hydrangea; the existing throwing technology has a certain positive effect on teaching, but it has shortcomings for high-level training and competition. The best shooting angle is 640 ≤ *α* ≤ 720, and the speed is 13.04 m/s ≤ *v*_0_ ≤ 13.70 m/s, which is a range of numerical matching between the two; the core problem of shooting technology is to shorten the shooting cycle and running distance through the cooperation of the best shooting angle and speed, so as to lay the foundation for improving the hit rate per unit time. *Suggestions*. Build national sports culture, improve the technical level, and promote the development of national sports to a higher level.

## 1. Research on the Origin of Hydrangea Throwing and Its Projection Technique

Throwing embroidered balls from the ancient weapon Feituo painted on the fresco of Huashan Mountain [1]. It can be seen from Figure 1(a) that the movement of throwing hydrangeas originated from the production and life of the ancient Zhuang people. It was used in war or hunting and was an effective weapon against distant targets (Figure 1(b)). The five-color bag recorded in the Song Dynasty “Xi Mancong Smile” as a way for young men and women in Zhuangxiang to express their love [2]. This sport has developed into today's traditional national sports with a history of more than 2000 years. He Weidong and Wu Guangjin have done a lot of in-depth studies on the history, culture, sports status, and competition rules of throwing embroidered balls [3]. Yang Qin and Yu Xiaoying et al. demonstrated that the best throwing angle = 65°, the best initial velocity *V*_0_=16.3 m/s, and the best passing point is the center of the passing circle [4–6]. The above research studies promote the inheritance of Hydrangea culture and the popularization and teaching of Hydrangea throwing, but they are all relatively common guiding thoughts and theories. It is of little significance to participate in the training and competition of high-level sports meeting, and it also hinders the competitive development of Hydrangea. At present, there is not a set of training method theory about the technique and tactics of high-pole throwing Hydrangea in China. The author set up the Hydrangea Team of Guangxi University of Science and Technology in 2015. After nearly a year of hard training and exploration, the author summed up a set of relatively mature technology and tactical theory of high-pole throw Hydrangea. After taking part in the 11th and 12th student Games of Guangxi, the author analyzes the existing problems of high-pole throwing Hydrangea from the technical level. The team won the gold medal of men's individual Hydrangea with high stroke, which proved the scientificity and reliability of the shooting technology with practice. The author hopes that these successful experiences can be continuously improved, improve the technical and tactical level of Hydrangea, and provide scientific and effective theoretical and practical reference for the training, competition, and teaching of Hydrangea in Colleges and universities, as well as the standardization and competitive development of Hydrangea.

## 2. Current Situation of Research on High-Pole Throwing Hydrangea Technology

### 2.1. The Function That Already Had Technology Theory Guides Practice

After consulting CNKI, it is found that there are few technical teaching, technical, and tactical training methods and theories on high-pole throwing Hydrangea. The best throwing angle = 65°. Among them, the most representative are the best initial velocity *V*_0_=16.3 m/s, and the best passing point is the center of the passing circle [4–6]. It is shown in Figure 2. These theories have a very good technical and theoretical guidance for the ball to pass the circle smoothly, but the prediction of the highest point of the ball, the falling point of the ball, and the next shooting situation is not enough, and the consideration is lack of coherence, so it is lack of guiding significance for high-level games. According to the rules of performance evaluation, the winner is the one with more hits per unit time. According to the dominant factors of competitive ability, high-pole shot Hydrangea belongs to the accuracy item of skill and mental ability [7]. According to the classification of action structure, it belongs to the fixed combination project of multiple action structure and has obvious periodic characteristics. Therefore, according to the rules of the game, we must complete more projection times in unit time and improve the hit rate in order to win the game, which is a test of athletes' psychology, skills, and physical fitness.

#### 2.1.1. Arc Height of the Highest Point of the Ball Flight

The best throwing angle and the best initial velocity are substituted into the formula *h*=*v*_0_sin  65°*t* − (1/2)*gt*^2^=16.3 × sin  65° × 1.5 − (1/2)*g*1.5^2^=10.75 m. When the ball is released from point O, the height from the ground is 2 m. When the ball flies the highest point A, the distance from OB is AE = 10.75 m, and the distance to the ground AC is 10.75 + 2 = 12.75 m.

When the air resistance is neglected, the rising and falling trajectory of the projected parabola are symmetrical to the left and right along the axis AE (Figure 2).

When the ball passes through the top of the arc and falls to point B 2 m above the ground, it forms a symmetrical arc trajectory with AE as the central axis with the projection point O. However, the actual landing point needs longer time and distance theoretically.

#### 2.1.2. The Horizontal Distance between the Ball and the Projection Point O When the Ball Falls to Point B 2 m above the Ground

*X*=*v*_0_cos  65°2*t*=16.3 × 0.42 × 3=20.54 m. This means that with the best angle and speed, the ball goes through the center of the circle and continues to fly until it reaches the top of the arc A, 12.75 m above the ground before falling. The horizontal distance OB between the symmetrical point B and the projection point at 2 m above the ground is OB = 20.54 m, while the actual landing point is farther. This representative projection technique can solve several situations of hand projection range and crossing circle, but the height of projection, landing time, and horizontal displacement increase, and the whole projection period is prolonged.

### 2.2. The Contradiction between Competition Rules and Existing Theories

Players can score points by throwing the Hydrangea over the pitching circle within the specified time. After each throw, they should run to the opposite pitching area to pick up their own ball and continue to throw the circle. The middle circle will get 1 point at a time. In this way, the players can repeatedly throw the ball in the two bowling areas. In the specified time, the number of shots in the middle circle will determine the merits and demerits [5]. As shown in Figure 2, from point O to point B to pick up the ball, he runs 20.54 − 14 = 6.54 m more than point D, which is 7 m away from the pole. To win the game by running back and forth in the shortest time, it is obviously not the most time-saving and physical method to increase the distance of 6.54 m each time to pick up the ball and run back.

The main mistakes in the above calculation are the ball passing through the center of the circle and reaching the maximum height at the same time are not considered and the coordination between the vertical component v0sin and the angle of release *α* is not analyzed. Take the formula *h*=*v*_0_2/2*g*, for example. The minimum release speed *v*_0_=14.3 m/s, and the maximum height of rising is ((14 × sin  650)(16 × sin  650)2/2*g*)=8.1 m; even if the ball passes through the circle from the center of the circle at 7.5 m, it will continue to rise 0.6 m and then fall, which will take longer time and increase horizontal displacement.

The above representative theory is lack of practicability for competition. The height of the arc top of the ball flying, the distance between the falling point and the projection point, the time and physical strength consumed by turning back and running back to the throwing line are not considered comprehensively. Therefore, with the best shooting height, angle, and speed, the result is not ideal. In addition, the best angle range *α*, velocity *v*_0_ range, and the matching of the two are not demonstrated.

## 3. Research and Practice Innovation of High-Pole Throwing Hydrangea Technology

### 3.1. The Assumption of Throwing Hydrangea

The player stands at the center line 7 m away from the pole. The longitudinal plane formed by the ball projection is directly opposite to the central axis of the pole. The air resistance is ignored. The ball is regarded as a particle and the circle is regarded as a coil without thickness. Because the game is to run back and forth in the shortest time to hit the shot to win, the top height *h* of the ball should not be too high, and the flying distance *x* should not exceed 14 m. The increase of vertical displacement *h* means more time consuming; the increase of horizontal displacement *x* means that the distance of running is extended, which consumes more physical strength and time. According to the principle of parabola symmetry, the top of the best arc should not exceed the circle. Assuming that the highest point of throwing is 10 m, it is the combination of the highest angle and speed to throw the ball from point O to point, a 10 m high from the level, and pass through the inner and lower edge of the circle. AB is the safe range of the upper edge of the projection (Figure 3). The falling point is close to the opposite side of the pole, which is conducive to saving time and physical strength. When the ball is thrown from the minimum angle to the bottom edge of the circle with a height of 9 m, it is the combination of the minimum speed and angle of the shot. Although the landing point is the farthest from point O (due to the symmetry principle, the landing site is near 14 m), due to the shorter flight time, it makes up for the lack of longer distance and also saves time and physical strength, which is conducive to creating excellent competition results.

### 3.2. Analysis of Three Cases of Ball Passing through Circle

#### 3.2.1. When the Highest Point of the Ball Passes through Point C at the Lower Edge of the Circle Which Is 9 m High from the Level

Horizontal displacement is

(1) $$\begin{array}{c} x=v_{0}\cos\;\alpha t. \end{array}$$

The time from vertical displacement *h* to circle lower edge and horizontal displacement 7 m is the same.

Therefore, *h*=(9 − 2)=(1/2)*gt*^2^, and the result is

(2) $$\begin{array}{c} v_{0}\cos\;\alpha =\frac{7}{\sqrt{14/g}}. \end{array}$$

Vertical displacement is *h*=*v*_0_sin  *α*(*t* − 1)/2*gt*^2^, and the result is

(3) $$\begin{array}{c} v_{0}\sin\;\alpha =\frac{\left(h+1/2gt^{2}\right)}{t=14/\sqrt{14/g}}, \end{array}$$

simultaneous with (1)–(3), (*v*_0_sin  *α*/*v*_0_cos  *α*)=tan  *α*=2, *α* ≈ 640, *v*_0_sin  *α*=*gt*, and the result is v_0_ = 13.04 m/s.

#### 3.2.2. When the Highest Point of the Ball Passes through Point B on the Upper Edge of the Circle 10 m from the Horizontal

*h* = 8, $t=\sqrt{16/g}$. Horizontal displacement is constant, and vertical displacement is $v_{1}\sin\;\alpha_{1}=\left(\left(h+1\right)/2gt^{2}\right)/t=\left(16/\sqrt{16/\text{g}}\right)$.

In the same way, (*v*_1_sin  *α*_1_/*v*_1_cos  *α*_1_)=tan  *α*_1_=16/7, and the result is *α* = 660 and v_1_ = 13.70 m/s.

#### 3.2.3. When the Ball Passes through Point A 10 m from the Horizontal and Passes through Point C at the Inner Lower Edge of the Circle

The sum of the ascent of 8 m to A and the fall of 1 m to C is equal to *h* = 7 m, *t*_2_ = (*t* + *t*_3_); then, $t_{2}=\left(\sqrt{16/\text{g}}\right)+\left(\sqrt{2/\text{g}}\right)$. Horizontal displacement is 7=*v*_2_cos  *α*_2_*t*_2_; then,

(4) $$\begin{array}{c} v_{2}\cos\;\alpha_{2}=\;\frac{7}{\left(\sqrt{16/g}+\sqrt{2/g}\right)}. \end{array}$$

The vertical displacement to A is 8=*v*_2_sin  *α*_2_*t* − (1/2)*gt*^2^; then, *v*_2_sin  *α*_2_*t*=8+(1/2)*gt*^2^.

Substitute $t=\sqrt{16/g}$; the result is

(5) $$\begin{array}{c} v_{2}\text{sin }\alpha_{2}=\frac{16}{\sqrt{16/\text{g}}}, \end{array}$$

simultaneous with (4) and (5), $\left(v_{2}\sin\;\alpha_{2}/v_{2}\cos\;\alpha_{2}\right)=\tan\;\alpha_{2}=\left(16/\sqrt{16/\text{g}}\right)/\left(7/\left(\sqrt{16/\text{g}}+\sqrt{2/\text{g}}\right)\right)=3.09$.

The result is *α* = 720 and v_2_ = 13.17 m/s. Substitute (4). Calculate the distance between the ball and point B at the top edge of the circle when it reaches the highest point A: *AB*=7 − *v*_2_cos  *α*_2_*t*; from (5), $v_{2}=\left(16/\sqrt{16/g}\right)\sin\;\alpha_{2}$, and *AB*=7 − 16(cos  *α*_2_/sin  *α*_2_)=1.80 m.

## 4. Result Analysis

Pitching over the circle can meet the needs of teaching, but it cannot meet the needs of high-level competition (Figure 4). The three situations of the ball passing through the circle are all parabola arc top does not exceed the circle, which is conducive to the saving of time and running distance, and can complete the shot more times, which is more conducive to improving the performance of the game.  Figure 5 shows the coach's projection demonstration.

1. When the highest point of the ball passes through the lower edge of the circle, the release angle is the lowest, *α* = 640, and the release speed is the lowest, *V* = 13.04 m/s. Although the distance between the falling point *D* and the projection point O is 14 m, the time is the shortest. It takes about 3 seconds from shooting to landing and rebounding to the highest point. After taking the shot, you can easily run to the opposite side, catch the rebound ball, and immediately turn around and throw it. Therefore, this combination of projection angle and speed does not waste time and extend the running distance, but in the three cases, it belongs to the fastest running requirement. Only by accelerating the speed can we grasp the ball and enter the next throwing cycle when the ball lands and rebounds, instead of bending down to pick up the ball and consume time and physical strength.
2. When the arc top of the ball is 10 m and falls through the inner and lower edge of the circle, the distance from the top of the arc to the top of the circle is 1.80 m, and the angle of release is the largest, *α* = 720. The speed of release is 13.17 m/s; less than this speed, the ball cannot pass through the circle, and higher than this speed, the ball will fall through the arc top E. Therefore, in the maximum angle of release, the speed should be large rather than small. Although the increase of height will prolong the time of falling, it is conducive to running and catching the ball calmly.
3. When the top of the ball passes through the upper edge of the circle, the angle of release is *α* = 660, and the velocity reaches the maximum value, *V* = 13.70 m/s. This is the combination of angle and speed, which is the farthest and takes the longest time among the three shooting methods. The distance between the landing point *D* and the projection point O is 14 m, which is the same as the first case in 3.1 above, but the time is longer, which is the time consuming for 8 m high falling.

## 5. Suggestions

- The top of the arc of the highest point of the trajectory of the projectile remains on the side of the projective side and does not exceed the circle. According to the symmetry principle, the falling point will be closer to the center of the rod, which is beneficial to shorten the running distance and reduce the physical consumption.
- The angle of the shot is better high than low because one cannot score a goal below 640 and the high angle can go into a circle in the falling process. When the release angle is 660, the maximum value of *V* = 13.70 m/s is taken as the boundary, and the projection speed *V* gradually decreases to 13.04 m/s when it goes down to 640 and to 13.17 m/s when it reaches 720.
- Constantly improve the technical and theoretical research level of Hydrangea throwing, promote the development of Hydrangea throwing and competition to a higher level, and provide theoretical and path reference for more national traditional sports to move from folk custom to competition, from leisure and entertainment to formal events, and develop into school sports and competitive sports, taking the development path of standardization and competition.

## Figures and Tables

**Figure 1:** Feituo rock painting in Huashan petroglyphs. (a) Huashan petroglyphs. (b) Feituo cliff painting.

**Figure 2:** The present best hand angle and speed matching diagram.

**Figure 3:** The best angle and speed matching diagram in practice.

**Figure 4:** Practice of high-pole throwing Hydrangea.

**Figure 5:** Coach demonstration.

## Data Availability

The datasets used and/or analyzed during the current study are available from the corresponding author upon request.
